# New insights into virulence mechanisms of rice pathogen *Acidovorax avenae* subsp. *avenae* strain RS-1 following exposure to *ß*-lactam antibiotics

This article has been retracted.

**DOI:** 10.1038/srep22241

**Published:** 2016-02-26

**Authors:** Bin Li, Mengyu Ge, Yang Zhang, Li Wang, Muhammad Ibrahim, Yanli Wang, Guochang Sun, Gongyou Chen

**Affiliations:** 1 State Key Laboratory of Rice Biology, Institute of Biotechnology, Zhejiang University, 310058, Hangzhou, China; 2 Department of Biosciences, COMSATS Institute of Information technology Sahiwal Campus, Sahiwal, Pakistan; 3 State Key Laboratory Breeding Base for Zhejiang Sustainable Plant Pest and Disease Control, Zhejiang Academy of Agricultural Sciences, Hangzhou 310021, China; 4 School of Agriculture and Biology, Shanghai Jiaotong University, Shanghai 200240, China

## Abstract

Recent research has shown that pathogen virulence can be altered by exposure to antibiotics, even when the growth rate is unaffected. Investigating this phenomenon provides new insights into understanding the virulence mechanisms of bacterial pathogens. This study investigates the phenotypic and transcriptomic responses of the rice pathogenic bacterium *Acidovorax avenae* subsp. *avenae* (Aaa) strain RS-1 to *ß*-lactam antibiotics especially Ampicillin (Amp). Our results indicate that exposure to Amp does not influence bacterial growth and biofilm formation, but alters the virulence, colonization capacity, composition of extracellular polymeric substances and secretion of Type VI secretion system (T6SS) effector Hcp. This attenuation in virulence is linked to unique or differential expression of known virulence-associated genes based on genome-wide transcriptomic analysis. The reliability of expression data generated by RNA-Seq was verified with quantitative real-time PCR of 21 selected T6SS genes, where significant down-regulation in expression of *hcp* gene, corresponding to the reduction in secretion of Hcp, was observed under exposure to Amp. Hcp is highlighted as a potential target for Amp, with similar changes observed in virulence-associated phenotypes between exposure to Amp and mutation of *hcp* gene. In addition, Hcp secretion is reduced in knockout mutants of 4 differentially expressed T6SS genes.

*Acidovorax avenae* subsp. *avenae* (Aaa) strain RS-1 has been reported to have strong virulence to rice plants^1^,^2^,^3^,^4^,^5^. One of the fundamental goals in the study of this rice pathogen is to identify virulence determinants during its interaction with the host^6^,^7^,^8^,^9^. Whilst the genome-wide transcriptomic response of strain RS-1 to *in vivo* infection of this rice pathogen has been examined with RNA-Seq previously^10^, in general, it is not easy to collect *in vivo* plant pathogenic bacteria, due to the contamination of plant tissues and low cell numbers in water. Therefore, an alternate method should be developed for genome-wide identification of virulence-associated genes in strain RS-1.

Recent studies have found that in addition to direct killing effect, exposure to antibiotics at sub-inhibitory concentrations could cause an increase or reduction in virulence of human and animal bacterial pathogens, while the pathogenic consequence of antibiotic resistance depends on the kind and concentration of antibiotics, as well as the tested bacterial strains^11^,^12^,^13^,^14^,^15^,^16^. Interestingly, a preliminary study revealed the naturally occurring *ß*-lactam-resistance of strain RS-1, which makes it necessary to examine the pathogenic consequence of β-lactam antibiotics exposure in this rice bacterial pathogen.

A number of studies have been performed to explore the underlying causes for the changes in virulence of human and animal bacterial pathogens when exposure to antibiotics^17^,^18^,^19^. In particular, differential expression of several genes encoding known virulence determinants has recently been proposed to be involved in bacterial virulence and antibiotic resistance^20^,^21^,^22^,^23^,^24^. However, little information was available about genome-wide analysis of gene expression under exposure to antibiotics, which will provide a comprehensive insight into molecular mechanisms of virulence in bacterial pathogen.

In this study, phenotypic changes and the genome-wide transcriptomic response of strain RS-1 were examined following exposure to *ß*-lactam antibiotics. The transcriptome was measured with RNA-Seq and validated by qRT-PCR using the primers listed in Table S1 and knockout mutations of the type VI secretion system (T6SS) genes. Secreted levels of the T6SS effector, Hcp, were measured by western blot analysis and ELISA, and its interaction with other T6SS components was investigated by using both a bacterial two-hybrid assay and a GST pull-down assay.

## Results

### Resistance to *ß*-lactam antibiotics

Growth of strain RS-1 was differentially affected by the three different *ß*-lactam antibiotics. At 48 h of exposure, there was no significant difference between with and without Amp in cell density with an OD600 of 1.20 and 1.24, respectively. In contrast, exposure to Amo caused a slight reduction in cell density with an OD600 of 0.97, while exposure to Pen resulted in a slight increase in cell density with an OD600 of 1.33 (Fig. 1a; Table S2).

### Changes in virulence-associated phenotypes

Biofilm formation was unaffected (*P* < 0.05) by the three different *ß*-lactam antibiotics after 48 h of adhesion (Fig. 1b). In contrast, swimming motility tests showed that exposure to Amp, Amo and Pen caused a 79.61%, 65.88%, and 51.76% reduction, respectively, in colony diameters (Fig. 1c). Furthermore, compared to the average FTIR spectrum of EPS from strain RS-1, exposure to Amp resulted in disappearance of one peak at 895.16 cm^−1^ representing phenyl ring substitution bands/alkenes (Figure S1). In addition, the emergence and height of seedlings were slightly reduced by Pen and Amo, but unaffected by Amp in the absence of pathogen (data not shown). Inoculation of strain RS-1 caused a 76.67%, 91.01% and 93.09% reduction in emergence, root length and plant height, respectively, compared to the negative control, while the virulence of strain RS-1 was unaffected by fusion of red fluorescent protein (*rfp*) (Fig. 2; Table S2). However, the virulence of strain RS-1 was attenuated under exposure to *ß*-lactam antibiotics especially Amp, which caused a 190.36%, 81.74% and 129.91% increase in emergence, root length and plant height, respectively, compared to the pathogen control (Fig. 2; Table S2).

The attenuation of virulence under exposure to Pen, Amp, and Amo was further justified by a significant (*P* < 0.05) decrease in root-colonization ability (Fig. 3). Indeed, exposure to the three *ß*-lactam antibiotics caused an 85.19–96.96% reduction in cell numbers of strain RS-1 and a 69.13–94.35% reduction in cell numbers of strain RS-1-*rfp* in rice roots. Furthermore, bacteria that were exposed to Amp were only sporadically observed on root surfaces, leaving the vascular bundle organization relatively intact. In contrast, in the absence of Amp, bacteria were widely distributed in both the inner and surface parts of root systems, which severely destroyed the vascular bundle structures of root cap, meristem and maturation zone (Fig. 3).

### Global transcriptomic profiling under exposure to Amp

The total number of reads obtained from each of the two samples under Amp (+) condition were 14,537,291 and 16,443,928, respectively, while the number of mapped cDNA reads were 12,679,967 and 15,732,263 per sample (Table S3, S4). Genome-wide transcriptomic analysis revealed that about 91% of the transcription profile of reads were assignable to the genome, and RNA-Seq data of the replicates showed high correlation, indicating good reproducibility (R = 0.98, *P* < 0.001; Fig. 4). RNA-Seq data under Amp (−) condition were obtained in our previous study^10^. The multidimensional scaling plot (MDS) shows less difference between two replicates within each individual, while great differences were observed between Amp (+) and Amp (−) (Fig. 4), indicating the response of strain RS-1 to Amp.

The 4851 genes are depicted on a smear plot or MA plot (Fig. 4), which is comparing observed and predicted relative expression values, and gives a snapshot of the combined consequences of variance in estimates. The points shown in the MA expression plot are a straightforward consequence of the fact that the measurements on each RNA-Seq have lower and upper bounds, and when they are differenced and averaged, these bounds translate into the seen linear constraints. Although the numerical values of these patterns appear to be substantially different from each other, the patterns exhibit certain similar structures in the parallel coordinate (PC) plots (Fig. 4). Obviously, we can see that an overlapped line is obtained and these special structures allow us to distinguish biclusters from unrelated expression values in the PC plot. Also, from these structures, we can predict the type of biclusters (Fig. 4).

### Differential gene expression

Genome-wide transcriptional analysis of differentially expressed genes in strain RS-1 under Amp (+) condition and their absolute and relative distributions of reads are described in Table S5. According to the method of Nagalakshmi *et al.*^25^, the transcript profile of the 4851 annotated genes was organized into four categories, while 809 genes (16.68%) had “high” levels of transcript profile, 1088 genes (22.43%) had “medium” levels of transcript profile, 2014 genes (41.52%) had “low” levels of transcript profile, and 940 genes (19.38%) were considered “not transcribed” under Amp (+) condition (Table S3).

Based on normalized gene expression values and RPKM ([reads/kb of gene]/[million reads aligning to genome])≥1, a Venn diagram reveals that 685 and 89 genes were specifically expressed under Amp (+) and Amp (−) conditions, respectively (Fig. 4; Table S5, S6). Among the 3226 commonly expressed genes under both conditions (Fig. 4; Table S7), 1496 differentially (more than 2-fold change and *P* value < 0.1) expressed genes including 1092 up-regulated genes (Table S8) and 404 down-regulated genes (Table S9) were identified at 2% probability level by using EdgeR^26^ and Cufflinks and TopHat v1.0.12^27^.

Interestingly, differential expression was also observed for those genes involved in *ß*-lactamase and T6SS. Indeed, among the 16 *ß*-lactamase-related genes predicted based on BLAST search in combination with retrieve of KEGG pathway database^28^ (Table S10), 2 genes and 1 gene was uniquely expressed under Amp (+) and Amp (−) conditions, respectively, while 8 genes including 7 up-regulated genes and 1 down-regulated gene were differentially expressed under Amp (+) vs. Amp (−) condition. Furthermore, 12 out of 21 T6SS genes were above 2-fold differentially expressed under exposure to Amp (Table S11). This indicated that these genes may be involved in the response of strain RS-1 to Amp.

### Functional categories of differentially expressed genes

A BLAST^29^ search based on cluster of orthologous group (COG)^30^,^31^ indicated that the 2270 unique and differentially expressed genes including 685 Amp (+), and 89 Amp (−) induced genes, as well as 1496 2-fold differentially expressed genes were sorted into 23 various functional groups, such as carbohydrate transport and metabolism (130), cell motility (71), defense mechanisms^22^, energy production and conversion (131), inorganic ion transport and metabolism (116), intracellular trafficking, secretion, and vesicular transport (54), secondary metabolites biosynthesis transport and catabolism (66), and signal transduction mechanisms (168) (Fig. 5; Table S5,6,7,8,9).

In addition to the COG search, classification with Gene ontology (GO)^32^ terms was also performed, which indicated that 1285 out of a total of 2270 unique and differentially expressed genes were mapped into 3 basic functional groups, Molecular Function (1400), Biological Process (753) and Cellular Component (296) (Table S12, Figure S2). The greater total number of genes in the three functional groups is due to that an annotated gene might be associated with one or more functional groups based on sequence homology.

### Validation of Illumina sequence data using qRT-PCR

Illumina sequence data were validated by comparing the gene’s total transcript level estimated from the RNA-Seq data with quantitative RT-PCR results of 21 selected T6SS genes in strain RS-1 (Table S11). The squared correlation coefficient r^2^ value between the two methods was 0.64 for Amp (+) vs. Amp (–) expression (Fig. 4). The high correlation observed in this study verified the efficiency and robustness of the RNA-Seq transcriptome of strain RS-1 cultivated under Amp (+) condition. This indicated that the above differentially expressed genes might be involved in the response of strain RS-1 to Amp. Notably, the expression of *hcp*, encoding a T6SS effector was more than 32-fold down-regulated under exposure to Amp (Figure S3a; Table S11), enabling further validation of the RNA-Seq data at the protein level.

### Validation of RNA-Seq data with ELISA and western blot of Hcp

The effectivity and sensitivity of the generated polyclonal antibody was validated by the positive reaction of dilutions up to 24000-fold with the purified overexpressed His-tagged Hcp protein of approximately 23 kDa, which was determined by both SDS-PAGE and western blot analysis (Fig. 6a). The dilution of 1/5000 was chosen for ELISA test and western blot, which showed that Hcp can be detected in 1.0 μg/ml of secretory, cytoplasmic, outer membrane and inner membrane proteins of strain RS-1. In contrast, Hcp was unable to be detected in 80 μg/ml extracted secretory proteins of strain RS-1 under exposure to Amp (Fig. 6b), suggesting a link between the presence of Amp and the reduction of secreted Hcp.

### Validation of RNA-Seq data by mutation and interaction of T6SS

In general, the *hcp*-mutant had a similar change in virulence-associated phenotypes such as virulence, growth, EPS composition and expression of T6SS genes with that exposure to Amp. At 48 h of incubation, mutation of *hcp* gene and exposure to Amp caused a slight reduction in cell density with an OD600 of 1.09 and 1.15, respectively (Fig. 1a,d,e). Mutation of *hcp* gene also caused the disappearance of one peak at 859.16 cm^−1^ based on FTIR analysis of EPS (Figure S1). Amp-induced changes in expression of T6SS genes were also observed in *hcp*-mutant, in particular, the expression of *hcp* gene was more than 676-fold down-regulated relative to the wild type (Figure S3b). Furthermore, Hcp protein could be detected in the cytoplasmic proteins of *lipo*-, *pppA*- and *impM*-mutants except *hcp*-mutant, but not in the secretory proteins of mutants of the four differentially expressed genes (Fig. 6c), demonstrating the importance of Hcp in the response of strain RS-1 to Amp. In addition, the Hcp was found to be able to interact with the other effector VgrG and other T6SS components such as Lipo *in vitro* using the bacterial two-hybrid and GST pull-down assays (Fig. 7a,b).

## Discussion

This study showed that bacterial growth and biofilm formation were unaffected after 48 h exposure to Amp. However, a difference was observed between with and without Amp in bacterial virulence, swimming motility, composition of EPS, and root-colonization ability. Furthermore, exposure to Amp resulted in differential expression of a large number of genes involved in bacterial virulence and antibiotics resistance based on genome-wide transcriptomic analysis of this rice bacterium by RNA-Seq. These results suggest that attenuation of virulence by exposure to *ß*-lactam antibiotics could provide an alternate strategy to identify new virulence determinants in bacterial pathogen.

The results presented here demonstrate the reliability of using strand-specific Illumina-based RNA-Seq for the transcriptomic studies of strain RS-1 cultivated under exposure to Amp. Comparative analyses revealed largely consistent global profiles for each RNA sample, regardless of sequencing depth, and a high percentage of the reads were assignable to the genome. Furthermore, the high correlation found between the biological replicates suggests a stable expression profile, which was verified by quantitative real-time PCR of the selected T6SS genes. Taken together, these results strongly indicate that our RNA-Seq data are reliable for further analysis of differential gene expressions.

Although the cut-offs between low, medium, and high transcript levels were arbitrary, there was a marked difference in the number of genes in each category between the presence and absence of Amp. This result was consistent with previous studies, which showed that bacteria adapt to antibiotics conditions by altering their patterns of gene expression^33^. The comparative transcriptomic analyses carried out here revealed a large number of genes that were differentially expressed under exposure to Amp.

Among the differentially expressed genes, particular focus was given to genes associated with *ß*-lactamase and T6SS. Exposure to Amp resulted in differential expression of 10 *ß*-lactamase-related genes, and a significant change in expression of T6SS genes. This is concordant with the results of Jones *et al.*^16^ and Knudsen *et al.*^34^, who found that sub-inhibitory concentrations of kanamycin were able to induce T6SS in *Pseudomonas aeruginosa*. Li *et al.*^10^ found that T6SS was involved in virulence of strain RS-1 based on the *in vivo* differential expression and the virulence loss of knockout mutants. These previous findings, coupled with our observations, suggest that the attenuation of virulence by exposure to Amp is associated with the differentially expressed T6SS genes.

This finding is further supported by comparing Amp susceptibility between the *hcp* deletion mutant and the wild type. No significant difference in the growth between the wild type and the *hcp* mutant was observed, and this observation is unaffected by the presence or absence of Amp. Even after 48 h of incubation, no change was observed. This highlights that whilst *hcp* gene has a role in virulence, it is unrelated to antibiotic resistance of strain RS-1.

In contrast with the down-regulation of the *in vivo* infection, most T6SS genes were up-regulated under Amp (+) condition. However, differential expression under both *in vivo* host infection and exposure to Amp highlights the involvement of these genes in the virulence of strain RS-1. Indeed, the differential expression pattern of T6SS genes between the above two conditions may be able to be well explained by the result that *in vivo* infection induced the virulence, but exposure to Amp attenuated the virulence of strain RS-1. Therefore, expression of most T6SS genes may be in general negatively associated with the virulence of strain RS-1.

Furthermore, response of strain RS-1 to Amp revealed by transcriptomic analysis was validated based on the qRT-PCR of T6SS genes. In particular, down-regulation of *hcp* gene expression was justified by a measured reduction in the secretion of effector Hcp, which was measured by ELISA and western blot using Hcp antibody. The expression change of effector Hcp both at the mRNA and protein levels highlights the importance of T6SS in response of strain RS-1 to Amp. In addition, a consistent change in the virulence-associated phenotypes was found between exposure to Amp and mutation of *hcp* gene by gene knockout in this study. This suggests that Amp may attenuate the virulence of strain RS-1 by targeting the T6SS, which has been reported to be involved in a widely variety of biological functions such as virulence, swimming motility, biofilm formation, colonization and antibiotics resistance^7^,^10^.

In contrast to the up-regulation expression of *impM*, *pppA* and *lipo* genes, the expression of *hcp* gene was down-regulated under exposure to Amp. This difference in expression pattern of T6SS genes may be mainly due to that *hcp* gene was directly involved in the secretion of effector Hcp, while secretion of effector was indirectly affected by the other three genes encoding structural proteins through the disruption of the T6SS machinery. Furthermore, this may partially explain the discrepancy between gene expression and gene function in this study, which indicated that mutation of the down-regulated gene *hcp* reduced the virulence of strain RS-1 to rice seedlings, while the virulence was differentially affected by the mutants of the up-regulated genes *pppA*, *lipo* and *impM*.

The role of Amp-induced differentially expressed genes in the attenuation of virulence was further justified by mutation analysis of T6SS genes. Indeed, our previous study revealed that the virulence of strain RS-1 was unaffected by the mutation of *pppA* and *lip* genes, but was reduced by the mutants of *hcp* and *impM* genes compared to the wild type. The discrepancy in virulence among the knockout mutants of four T6SS genes revealed the complexity in the role of T6SS in bacterial virulence. The loss in virulence of the mutants may not be due to each T6SS gene itself, but may be more likely due to an indirect disruption in structure of the T6SS machinery, functioned as a whole in influencing the secretion of effector proteins, eventually resulting in the change in a variety of biological functions such as the loss of virulence^10^.

This study revealed that T6SS effector Hcp protein was unable to be detected in the secretory proteins of *lipo*-, *impM*-, *pppA*- and *hcp*-mutants, indicating that these genes were involved in the secretion of Hcp. Therefore, the reduction in virulence of *hcp*- and *impM*-mutants may be mainly due to the reduction of Hcp secretion. The reduction in Hcp secretion but not in virulence of *pppA*- and *lipo*-mutants may be at least partially attributed to the increased secretion of the other effectors such as VgrG, which could be justified by the interaction of Hcp with both Lipo and VgrG in this study using both a bacterial two-hybrid assay and a GST pull-down assay.

In summary, Amp-induced changes in virulence-associated phenotypes were validated by the RNA-Seq data, which revealed differential expression of a large number of genes in particular many important virulence-associated genes such as T6SS genes under Amp (+) condition, while the role of differentially expressed T6SS genes in virulence was justified by the reduced secretion of effector Hcp from the four constructed T6SS mutants. Furthermore, the inconsistence between the reduction of Hcp secretion and the loss of virulence for knockout mutants of T6SS genes may be mainly due to the involvement of the other T6SS effectors such as VgrG. In contrast with the role in virulence, T6SS effector Hcp seems not to be responsible for Amp resistance in strain RS-1. Overall, this study clearly indicated that RNA-Seq-based transcriptome analysis of the rice pathogenic bacterium under exposure to Amp produced a robust, sensitive, and accessible data set for identification of novel virulence-associated genes in bacterial pathogen.

## Methods

### Bacteria, antibiotics and plasmids

Bacterial strains and plasmids utilized in this study were listed in Table 1. *Escherichia coli* (*E. coli*) strains and Aaa strains were routinely cultured in Luria-Bertani (LB) medium at 37 °C and 30 °C, respectively. Stock solutions of 100 mg/ml were prepared by dissolving Kanamycin and *ß*-lactam antibiotics Ampicillin (Amp), Penicillin G (Pen) and Amoxicillin (Amo) (Bio Basic Inc., Canada) in sterile ddH_2_O.

### Bacterial growth under exposure to *ß*-lactam antibiotics

The growth of strain RS-1 under exposure to different *ß*-lactam antibiotics was evaluated by inoculating 5 μl overnight cultures into 5 ml of LB broth and then adding stock solutions of antibiotics to obtain the final concentrations of 100 ng/ml, while the control was added using the same volume of sterile water. Bacterial numbers were determined by measuring the OD600 using a Thermo Multiskan EX Micro plate Photometer (Perkin Elmer Lambda 35 UV/VIS, Thermo Fisher Scientific Inc., USA) after incubation at 180 r/min, 30 °C, for 0, 6, 12, 24, and 48 h, respectively.

### Measurement of virulence-associated phenotypes

Changes in virulence-associated phenotypes under exposure to *ß*-lactam antibiotics were determined as follow. In brief, assays of biofilm formation and swimming motility were performed as described by Liu *et al.*^35^, while pathogenicity to rice seedling was carried out based on the method of Li *et al.*^1^. Root colonization assay was performed as described by Chen *et al.* 36,37 with minor modification. Germinated rice seeds were bacterized for 48 h using strain RS-1-*rfp*, which was constructed by fusing the *rfp*-containing expression vectors pBBR (N-terminal RFP) into strain RS-1 using pulse cell transformation (GenePulser Xcell, BIO-RAD, USA). Bacterial colonization on root in 3.0 cm of length was observed using fluorescence microscope (Leica DMIRB, Germany), while bacterial numbers were counted based on plate count method as described by Kutter *et al.*^38^. Extraction and FTIR analysis of bacterial EPS were performed as described by Patel *et al.*^39^ and Ge *et al.*^40^, respectively.

### RNA-Seq and data analysis

After 48 h incubation under exposure to Amp of 100 μg/ml, total RNA extraction and purification were performed using High Pure RNA Isolation Kit (ROCHE, USA). Concentrations of the purified RNAs were calculated by measuring absorbance at 260 nm using Nanodrop 2000 C (Thermo Fisher Scientific, Maryland, USA). Furthermore, RNA-Seq library generation, Illumina HiSeq 2000 Sequencing, and data assembly and annotation as well as differential gene expression analysis were performed following the alignment with the genome of the reference strain ATCC 19860 (Accession Number CP002521) by using Degust, a web tool consisting of a backend that uses limma^41^ and edgeR^26^ to perform statistical analysis, and a dynamic frontend for the interactive visualization (http://www.bioinformatics.net.au/) and EDGE-pro^42^.

### Consistency of qRT-PCR with RNA-Seq profile

Genome-wide transcriptomic profile of strain RS-1 under exposure to Amp was further validated by qRT-PCR of the 21 selected T6SS genes, while 16 S rRNA gene was used as the reference. Primers design, total RNA extraction, the cDNA synthesization, qRT-PCR, and the correlation analysis between the two methods were conducted as described in our previous study^10^.

### Secretion of T6SS effector Hcp under exposure to Amp

The full-length *hcp* with *BamH* I and *EcoR* I restriction sites was amplified by the designed primer pair Pt-hcp, and cloned into pET-28a^+^to construct the expression plasmid pET-28a^+^-*hcp*, which was transferred into *E. coli* BL21 (DE3) for expression of Hcp-His fusion protein. Total proteins were extracted based on the method of Lin *et al.*^43^. After purification over a Ni-NTA-Sepharose column (Bio Basic Inc., Canada), separation by a 15% SDS-PAGE gel and confirmation by western blot using Anti-6 × His Tag rabbit polyclonal antibody as described by Yang *et al.*^44^, the Hcp-His fusion protein was used for the immunization of rabbits to obtain polyclonal antisera. Following the examination of the sensitivity and specificity, the polyclonal antisera at a 1:5000 dilution was used for detection of Hcp by indirect ELISA^45^ and western blot analysis.

### Hcp secretion and characterization of T6SS mutants

The role of Hcp in bacterial response to Amp was examined by measuring biofilm formation, swimming motility, pathogenicity and EPS composition of the *hcp*-mutant as described above. In addition, the polyclonal antisera was used for detection of Hcp from cytoplasmic and secretory proteins in knockout mutants of differentially expressed T6SS genes *hcp, lipo, pppA* and *impM*, which were constructed based on the method of Penfold and Pemberton^46^. In brief, the internal DNA fragment was amplified with the corresponding primers listed in Table S1. The resulting fragment was ligated into the suicide vector pJP5603. After replication and proliferation in *E. coli* S17-1 λ pir, the recombinant plasmid was introduced into strain RS-1 via electroporation. The pathogenicity of these mutants to rice seedlings was determined as described by Li *et al.*^10^.

### Interaction of effector Hcp with T6SS VgrG or Lipo

Bacterial two-hybrid assays were performed by mixing both recombinant plasmids pCH363-*hcp* and pKNT25- (*vgrG* or *lipo*) well and then co-transferring into reporter strain BTH101 as described by Chen *et al.*^36^,^37^. The former recombinant plasmid was generated by amplifying the full-length *hcp* using primer Th-hcp (Table S1), digesting with BamH I/EcoR I, and cloning into the pCH363, while the latter recombinant plasmid was generated by amplifying the full-length *vgrG* or *lipo* using primers Th-VgrG and Th-lipo, respectively, and then fusing into pKNT25 after digestion with Xba I/EcoR I and BamH I/EcoR I, respectively.

GST-pull down assay was carried out by incubating equal amounts of the fusion proteins Hcp-GST and VgrG-His (or Hcp-His and Lipo-GST). The primers of Pt-hcp, Th-vgrG, Th-hcp and Th-lipo were used to amplify the full-length *hcp, vgrG* and *lipo* for the construction of recombinant plasmids, which were induced into *E. coli* BL21 (DE3) cells for expression of the VgrG-His, Hcp-His, Hcp-GST and Lipo-GST. The fusion protein with GST tag was purified using GST-Sepharose 4B beads (Bio Basic Inc., Canada), while the fusion protein with His-tag was purified as described above. Western immunoblotting was performed as described above.

### Statistical analyses

The software STATGRAPHICS Plus, version 4.0 (Copyright manugistics Inc., Rockville, Md., USA) was used to perform the statistical analyses. Levels of significance (*P* < 0.05) of main treatments and their interactions were calculated by analysis of variance after testing for normality and variance homogeneity.

## Additional Information

**Accession codes:** RNA-Seq raw data files are accessible through the GEO Series accession number-GPL17669: GSM1220690-*In vitro* Rep 1; GSM1220691-*In vitro* Rep 2; accession number-GSE68734: GSM1679892-Amp Rep 1; GSM1679893-Amp Rep 2.

**How to cite this article**: Li, B. *et al.* New insights into virulence mechanisms of rice pathogen *Acidovorax avenae* subsp. *avenae* strain RS-1 following exposure to β-lactam antibiotics. *Sci. Rep.* **6**, 22241; doi: 10.1038/srep22241 (2016).

## Supplementary Material

Supplementary Information

Supplementary Table S4

Supplementary Table S5

Supplementary Table S6

Supplementary Table S7

Supplementary Table S8

Supplementary Table S9

Supplementary Table S10

Supplementary Table S11

Supplementary Table S12

## Figures and Tables

**Figure 1:** Changes in virulence-associated phenotypes of *Acidovorax avenae* subsp. *avenae* strain RS-1 under exposure to *ß*-lactam antibiotic and mutation of *hcp* gene. (**a**) Growth of the *hcp*-mutant and the wild type in the presence and absence of Amp; (**b**) Biofilm formation under exposure to *ß*-lactam antibiotic; (**c**) Motility under exposure to *ß*-lactam antibiotic; (**d**) Biofilm formation of the *hcp*-mutant; (**e**) Motility of the *hcp*-mutant. The same letters indicate there are no significant differences (*P* < 0.05) among treatments. Each treatment had eighteen replicates and this experiment was repeated three times independently with similar results.

**Figure 2:** Pathogenicity of *Acidovorax avenae* subsp. *avenae* strain RS-1 to rice seedlings. (**a**) Exposure to Amp; (**b**) Mutation of *hcp* gene. Briefly, rice seeds were immersed into bacterial suspension of approximately 10^8^ CFU/ml for 2 h at room temperature, then sown in commercial pots filled with perlites in greenhouse at 30 °C in the daytime and 24°C in the night. Bacterial virulence was determined by measuring the germination rate of rice seeds after 10 d of sowing. Control seeds were treated by ddH_2_O. Each pot contains 10 seeds. *rfp* (−): strain RS-1 without *rfp*; *rfp* (+): strain RS-1 harbored a constitutively expressed *rfp* reporter fusion gene. The same letters indicate no significant difference (*P* < 0.05) among treatments. Each treatment contains three pots, while this experiment was repeated independently three times with similar results.

**Figure 3:** Root colonization of *Acidovorax avenae* subsp. *avenae* strains RS-1 and RS-1 + *rfp* under exposure to *ß*-lactam antibiotic. (**a**) Root colonization of strain RS-1 + *rfp* under exposure to Amp; (**b**) Cell numbers of strain RS-1 under exposure to *ß*-lactam antibiotics; (**c**) Cell numbers of strain RS-1 + *rfp* under exposure to *ß*-lactam antibiotics. Root colonization assay was conducted as described by Chen *et al.* (2012)^36^,^37^ using strain RS-1 + *rfp*, which was constructed by fusing the *rfp*-containing expression vectors pBBR (N-terminal RFP) into strain RS-1 using pulse cell transformation (GenePulser Xcell, BIO-RAD, USA). Surface sterilization, bacterization and sowing of the germinated rice seeds were performed as described above. After the length of rice roots reached about 3.0 cm, bacterial colonization on root surfaces was determined by observing the express of the red fluorescent proteins using a fluorescence microscope (Leica DMIRB, Germany). Seedlings without bacterial inoculation were used as the control. The harvested roots were washed three times in sterilized PBS buffer to remove unattached cells. Colony number per g fresh sample was counted based on the plate count method as described by Kutter *et al.*^38^. The experiment was repeatedly twice, and the representative results were shown (n = 6). The same letters indicate no significant differences (*P* < 0.05) among treatments.

**Figure 4:** Analysis of RNA-Seq data including both Amp (−) data obtained from Li *et al.* (2014)^10^, and Amp (+) data determined in this study. (**a**) Principle component analysis of RPKM-based expression values of *Acidovorax avenae* subsp. *avenae* strain RS-1 transcriptome under Amp (+) and (−) conditions. The 4 samples shown in the 2D plane spanned by their first two principal components. This type of plot is useful for visualizing the overall effect of experimental covariates and batch effects. For this data set, no batch effects besides the known effects of condition and lib Type are discernible; (**b**) Multi-dimensional scale plot of Amp (+) and (−) based on RNA-Seq data. Dimension 1 and dimension 2 separate all 4 RNA-Seq libraries based on the expression value of the genes that passed all data filtering criteria prior to differential gene expression analysis; (**c**) Venn diagram representing the number of differentially expressed genes in strain RS-1 under Amp (−) (blue circle) and Amp (+) (yellow circle) conditions; (**d**) DEGseq2 comparisons are presented in MA-plots which shows genes are differentially expressed under Amp (+) vs. Amp (−) condition. A cutoff of *P*-value < 0.01 (Benjamini Hochberg method or “FDR”) was chosen. Each dot represents an STG. Red dots represent statistically significantly differentially expressed genes; (**e**) The PC plots of gene expression data under Amp (+) and (−) conditions; the constant bicluster shows an overlapped line across all the columns where the number of overlapped lines is determined by the number of rows, the constant row bicluster shows zero slope lines across all the columns where the number of lines is again determined by the number of rows, and the constant column bicluster shows an overlapped non-zero slope line across all the columns; (**f**) Correlation (R = 0.95–0.98, *P* < 0.001) of RNA-Seq data between two biological replicates of strain RS-1 under Amp (+) condition; (**g**) The correlation between RNA-Seq expression data (log_2_) and qRT-PCR data (log_2_) (*P* < 0.001, r^2^ = 0.64).

**Figure 5:** Classification of significantly differentially expressed genes under Amp (+) vs. Amp (−) condition of *Acidovorax avenae* subsp. *avenae* strain RS-1 transcriptome based on designation of COG.

**Figure 6:** Secretion of T6SS effector Hcp in *Acidovorax avenae* subsp. *avenae* strain RS-1 under exposure to Amp and mutation of T6SS genes. (**a**) Hcp detection in four different components using polyclonal anti-Hcp rabbit serum generated by Huaan company (Hangzhou, China) using Hcp-His fusion protein (about 23 kDa), which was obtained by amplification of *hcp* gene (483 bp) using the designed primers (Table S10), digestion with both BamH I and EcoR I, and ligation to plasmid pET-28a, overexpression by IPTG induction in *Escherichia coli* BL21 (DE3), purification using Ni-NTA-Sepharose Beads (Sangon Biotech, China), and size-fractionated on a 15% SDS-PAGE gel as described by Yang *et al.*^44^. The tested proteins including Hcp-His fusion protein were subsequently validated by western blot and ELISA analysis. Western blot was performed using primary polyclonal antibody (1:5000) followed by a secondary antibody using Horseradish Peroxidase-Conjugated goat anti-rabbit immunoglobulin G (Sangon Biotech, China), and then visualized using ImageQuant LAS 4000 (GE Health). The indirect ELISA was performed according to the method of Slutzki *et al.*^45^ by coating each well in the immunoassay plates (Maxisorp, Nunc, Denmark) using 1.0 μg/ml of the tested proteins, charging with rabbit poly-antibody at a dilution of 1:5000 according to the protocol of EL-TMB colored reagents (Sangon Biotech, China), and then measuring the OD 450 nm value in an ELISA reader (Multiscan Ex. Lab systems, Thermo Fisher Scientific Inc., USA). M: marker; IM: inner membrane; OM: outer membrane. (**b**) ELISA detection of Hcp from secretory proteins using polyclonal antibody (1:5000) under Amp (+) condition. (**c**) ELISA detection of Hcp from cytoplasmic proteins and secretory proteins in T6SS mutants using polyclonal antibody (1:5000). The purified Hcp-His fusion protein of 1.0 μg/ml was used as the positive control, while the BSA was used as the negative control. Each experiment was repeated three times independently with similar results.

**Figure 7:** Interaction of T6SS VgrG and Lipo with Hcp effector *in vitro* (**a**) Bacterial two-hybrid assay; (**b**) Pull-down assay; (**c**) Specificity of antibody. Each experiment was repeated four times independently with similar results.

**Table 1:** Strains and plasmids applied in this study.

Strain or plasmid	Relevant characteristics	Source or reference
Strains		
* Acidovorax avenae* subsp. *avenae* RS-1	Amp^R^; The pathogen of bacterial brown stripe of rice, isolated from the diseased rice from Zhejiang province in China	Lab collection
* Acidovorax avenae* subsp. *avenae* RS-1-*rfp*	Amp^R^, Kan^R^; The recombinant *Acidovorax avenae* subsp. *avenae* RS-1, contains a pBRM plasmid with a red fluorescent protein.	This study
* hcp* mutant strain Δ*hcp* of *Acidovorax avenae* subsp. *avenae*	Amp^R^, Kan^R^; The *hcp*-mutant of *Acidovorax avenae* subsp. *avenae* RS-1	This study
* Escherichia coli* DH5α	F-Φ80d lacZΔM15Δ (lacZYA-argF) U169 recA1 endA1, hsdR17(rk–, mk+) phoAsupE44 λ– thi-1 gyrA96 relA1	Invitrogen
* Escherichia coli* S17-1 λ *pir*	λ Lysogenic S17-1 derivative producing π protein for replication of plasmids carrying oriR6K; recA pro hsdR RP4-2-Tc::Mu-Km::Tn7 λ– pir	Penfold and Pemberton (1992)^46^
* Escherichia coli* BTH101	Host for overexpressing proteins in bacterial two-hybrid	Chen *et al.*^36^,^37^
* Escherichia coli* BL21(DE3)	Host for overexpressing proteins driven by T7 promoter	Invitrogen
Plasmids		
* *pBBR	Kan^R^; broad host expression vector	CAU
* *pBRM	Kan^R^; recombinant broad host expression vector with *rfp*	CAU
* *pJP5603	Kan^R^; R6K-based suicide vector; requires the pir-encoded π protein for replication	Penfold and Pemberton (1992)^46^
* *pGEM-T	Amp^R^; cloning vector	Promega
* *pET-28a^+^	Kana^R^; expression vector with His label	Promega
* *pGEX-6p-1	Amp^R^; expression vector with GST label	Promega
* *pET-28a^+^-*vgrG*	Kana^R^; recombinant expression vector with His label and a *vgrG*	This study
* *pGEX-6p-1-*hcp*	Amp^R^; recombinant expression vector with GST label with a *hcp*	This study
* *pGEX-6p-1-*lipo*	Amp^R^; recombinant expression vector with GST label with a *lipo*	This study
* *pCH363	Amp^R^; expression vector for bacterial two-hybrid test	Chen *et al.*^36^,^37^
* *pKNT25	Kan^R^; expression vector for bacterial two-hybrid test	Chen *et al.*^36^,^37^
* *pCH363-*hcp*	Amp^R^; recombinant expression vector for bacterial two-hybrid test	This study
* *pKNT25-*lipo*	Kan^R^; recombinant expression vector for bacterial two-hybrid test	This study
* *pKNT25-*VgrG*	Kan^R^; recombinant expression vector for bacterial two-hybrid test	This study

aAmp^R^: Ampicillin resistance; Kan^R^: Kanamycin resistance; CAU: China Agricultural University.
